This article has been retracted.

# Apelin Receptor (APJ) Expression during Cardiopulmonary Bypass in Children Undergoing Surgical Repair

**DOI:** 10.1371/journal.pone.0106262

**Published:** 2014-09-03

**Authors:** Susan Walker, Mark H. D. Danton, Alexander D. Lang, Fiona Lyall

**Affiliations:** 1 Institute of Medical Genetics, University of Glasgow School of Medicine, Royal Hospital for Sick Children, Glasgow, United Kingdom; 2 Department of Paediatric Cardiac Surgery, Royal Hospital for Sick Children, Glasgow, United Kingdom; University of Bristol, United Kingdom

## Abstract

**Background and Aims:**

In human adults, and animals, the Apelin-APJ ligand-receptor system is emerging as having a role in the pathogenesis of cardiovascular function and heart failure. The aim was to investigate expression, and regulation by oxygen, of the Apelin APJ receptor (APJ) in myocardium obtained from children undergoing corrective surgery with cardiopulmonary bypass for repair of congenital heart defects.

**Methods:**

Western blotting and Real-time PCR were used to determine if APJ was expressed in the infant myocardium, if expression was influenced by the duration of myocardial ischemia and if any relationship existed between APJ expression and early post-operative outcome. The next aim was to determine if there was a difference in mRNA expression of APJ in myocardium from cyanotic patients compared with acyanotic patients and if re-perfusing myocardium *in vitro* with either hypoxic, normoxic or hyperoxic oxygen affected APJ mRNA expression.

**Results:**

APJ was expressed in all myocardial samples and myocardium exposed to longer durations of ischemia and cardioplegia expressed higher levels of APJ (p<0.05). There was a significant correlation between APJ expression in myocardium resected after 10 min with both oxygen extraction ratio (p = 0.021, rho = −0.523) and mixed venous oxygen saturation (p = 0.028, rho 0.52). This association did not exist for myocardium collected before 10 min. There was no difference in APJ expression between cyanotic and acyanotic patients. No difference was found in APJ expression whether re-perfused with low, normal or high oxygen.

**Conclusions:**

Changes in APJ expression were observed during cardiopulmonary bypass in children and the reasons for this require further investigation.

## Introduction

Tetralogy of Fallot (TOF) is the most common cyanotic congenital heart disease. TOF is characterized by the presence of ventricular septal defect, pulmonary stenosis, aortic over-ride and right ventricular hypertrophy. Complete repair is performed in infancy and is associated with a low mortality risk (<2%) [1]. Post-operative right ventricle (RV) dysfunction is common and impacts on early patient outcome. In the decades that follow TOF repair continuing RV dilation and dysfunction can limit exercise capacity and life expectancy. The etiology of RV dysfunction post TOF correction is multifactorial. Prior to surgery the RV myocardium is perfused with blood of reduced oxygen content (cyanosis) and the ventricle is pressure loaded due to the presence of the VSD. At the cellular level the effects include hypertrophy, a chronic mismatch of oxygen supply and demand, apoptosis, matrix remodeling and fibrosis [2].

In the use of cardiopulmonary bypass (CPD), required in the repair of TOF, the myocardium is exposed to three phases of perfusion: (a) an initial high oxygen tension/supra-physiological perfusion, (b) ischemia during cross clamp and (c) further reperfusion. Despite use of cardioplegic techniques that induce myocardial electromechanical cessation during the ischemic-cross clamp phase, myocardial ischemic-reperfusion occurs. Whether the chronically hypoxic (cyanotic) myocardium is more or less tolerant of CPB related injury compared to non-cyanotic patients is unclear but the limited literature supports the latter.

Apelin is the ligand for the G protein-coupled APJ receptor [3], [4]. The APJ receptor has been shown to counteract damaging effects of angiotensin II [5]. Other actions include regulation of fluid and glucose homeostasis, vessel formation, inhibition of vasopressin release, regulation of vascular tone, decreases blood pressure and increases diuresis as well as playing a role in diabetes and obesity [6]. The APJ receptor is expressed in endothelial cells, vascular smooth muscle cells and cardiomyocytes [7]. The main source of Apelin is the heart [8] and the primary function of the Apelin-APJ receptor system is thought to be in the cardiovascular system [9]. Within the myocardium itself, Apelin-APJ activation increases contractility of myocardiocytes and is one of the most powerful positive inotropes known [10]. Apelin functions as a potent vasodilator [11], [12] mediated through NO dependent pathways of vasodilatation [13]. To date, the APJ receptor system has not been investigated in the infant myocardium or indeed in the context of open-heart surgery for correction of TOF. In part the reason for this is the extreme difficulty in obtaining infant myocardial tissue, the very small size of tissues samples and the lack of collaborative basic science with the clinical interface.

The first aim of this study was to determine if the APJ receptor was expressed in the infant myocardium and if there was any differences in APJ receptor protein expression in myocardium resected at the onset of surgery compared to myocardium resected further into the surgical time and which had been exposed to a longer ischemic time. The second aim was to determine if expression of the APJ receptor was related to clinical parameters relevant to cardiac physiology (listed in Table 1). The next aim was to determine if there was a difference in mRNA expression of the APJ receptor in myocardium resected from cyanotic patients compared with control acyanotic patients (sub-aortic stenosis or truncus arteriosus patients) after 15–30 min of cross-clamp time when a effect of ischemia on APJmRNA might be observed. The final aim was to re-perfuse resected myocardium, *in vitro*, with either hypoxic, normoxic or hyperoxic oxygen concentrations and determine the effects on APJ mRNA receptor expression.

**Table 1:** Peri-operative characteristics of the patients studied for APJ protein analysis.

Patient details (n = 20)	Median (inter-quartile range)
Age (months)	19 (6.8–24.3)
Gender (number)	11 males
Weight (kg)	9.9 (7.9–12.2)
Haematocrit level (%)	42.5 (40.8–50.0)
Pre-op O_2_ saturation (%)	89 (68–97)
Prior BT Shunt (number)	8
**PRE-OP ECHO**	
RV wall thickness (cm)	0.70 (0.57–0.83)
IVS wall thickness (cm)	0.76 (0.54–0.94)
Sm–tricuspid annulus (cm/s)	8.92 (7.28–11.55)
Sm–basal septum (cm/s)	4.86 (3.73–6.10)
Sm–mitral annulus (cm/s)	4.86 (3.33–6.23)
Cross clamp time (min)	84 (61.8–130.0)
Bypass time (min)	84 (61.8–130.0)
**POST-OP ITU Parameters**	
Troponin-I (ng/mL)	14.5 (7.6–51.0)
Inotrope score	10.25 (0.8–16.3)
Haemoglobin (g/dL)	11.8 (10.4–14.0)
SvO_2_ (%)	66 (55.5–71.3)
Oxygen extraction ratio	0.33 (0.28–0.42)
Lactate	1.4 (0.88–1.9)
Ventilation time [hours]	111 (58.7–195.2)
Critical care stay [days]	111 (58.7–195.2)
**ECHO Day 1**	
Sm–tricuspid annulus (cm/s)	3.8 (2.50–4.77)
Sm–basal septum (cm/s)	2.96 (2.13–4.48)
Sm–mital annulus (cm/s)	4.59 (3.61–6.46)

All data expressed in median (interquartile range). BTS Blalock–Taussig shunt, IVS interventricular septum, Sm systolic myocardial velocity, XC (cross clamp), SvO_2_ mixed venous oxygen saturation.

## Materials and Methods

### Ethics

Ethical approval for this project was given by the Greater Glasgow and Clyde Health Board. The study complies with the Declaration of Helsinki. Parents were provided with information sheets approved by the ethics board to inform them about the study prior to given signed written consent on the day their child underwent surgery. Due to the small amount of tissue resected at surgery, and thus available for research, different patients were recruited to for each set of experiments as outlined below. Power calculations were performed to ensure sufficient patients were used in each group as shown previously [14]. The study was performed over a three year period in order to be able to recruit sufficient patient numbers.

### Perioperative tissue Doppler echocardiography

Tissue Doppler echocardiography was performed under general anaesthesia as described previously [14] before skin incision and repeated on post-operative day 1 in the intensive care unit (ICU) and then 1 week later. Pulsed wave tissue Doppler velocity measurements at the tricuspid annulus, basal septum and mitral annulus were obtained from an apical four-chamber view to quantify systolic myocardial velocity. Three or more loops were stored for subsequent offline analysis. The presence of restrictive right ventricle physiology was defined as antegrade flow across the pulmonary artery coincident with atrial systole in all respiratory cycles (parasternal short axis right ventricle outflow tract view) [15].

### Surgical repair and myocardial protection

Standard repair was performed as described previously [14] by ventricular septal defect (VSD) closure and resection of RV infundibular muscle via transtricuspid and transpulmonary routes using moderate hypothermia and blood cardioplegia. Prior to cardiopulmonary bypass, all patients received oxygen supplementation and fractional inspired oxygen was adjusted to maintain adequate oxygenation whilst avoiding hyperoxia. Post-repair Epicardial echo was routinely performed to exclude any residual lesion at the end of the procedure. Direct RV and left ventricle pressures were measured intra-operatively post-repair.

### Chemicals and reagents

All chemicals and reagents were purchased from Sigma-Aldrich (U.K.) unless stated otherwise. Supplemented media for tissue culture was Medium 199 (Sigma, M4530-100ML) containing 5% fetal bovine serum (Sigma, F9665) and 1% antibiotic antimycotic solution. (Sigma A5955).

### Patients for Western blot experiments

Twenty patients with TOF who underwent surgical repair at the Royal Hospital for Sick Children, Glasgow were recruited. The clinical details of the patients are shown in Table 1. A separate control group of age-matched children (*n* = 15) presenting with an innocent murmur (median age, 27.1; inter-quartile range, 4.0–47.2 months versus TOF patients; *p* = 0.62) was recruited to obtain normal reference values for tissue Doppler myocardial velocities [14].

### Tissue collection for Western blot analysis

All myocardium resected from the RV outflow tract, as part of the surgical repair, was collected for protein analysis. Muscle was snap-frozen immediately in liquid N_2_ following resection and stored at −70°C until required. Pieces of muscle were grouped according to the ischemic time point at collection as follows. The beginning of myocardial ischemic time was defined as the time when aortic cross-clamp was applied and the first dose of cardioplegia infused. The ischemic baseline period was defined as <10 min after aortic cross-clamp and before further repeated cardioplegia administration. This group of myocardial samples was represented as close to the pre-operative APJ receptor expression in the myocardium as possible and is referred to herein as (<10 min). The 10 min time also allowed sufficient tissue to be collected in both experimental groups. Subsequent muscle samples resected after this period, referred to as >10 min, were grouped together. Comparison of the two groups would allow any effect of ischemic time of surgery on APJ receptor expression. Due the tiny amounts of tissue available it was not possible to divide the time points any further.

### Western Blot Analysis

Western blotting and protein transfer was performed as described previously^16^ with some modifications. Fifty µg of each sample was separated on 10% sodium dodecyl sulfate-polyacrylamide resolving gels. The APJ antibody (rabbit polyclonal, Phoenix Pharmaceuticals) was used at a concentration of 1/1000. Membranes were washed and then incubated for 1 h at RT with horseradish peroxidase conjugated donkey anti-rabbit secondary antibody (Abcam) diluted to 1∶1000. The same sample aliquots were detected with an HSP 70 antibody to ensure even protein loading; we have previously shown that HSP 70 is constitutively expressed in these same samples taken from the same patients [14]. Immunologically reactive proteins were visualised and quantified as described previously [16]. We previously confirmed that scanning densitometry provided similar results to other quantitative methods [16]. Care was taken to ensure that the bands which were scanned fell on the linear range of protein loading as described previously [16]. Since several gels were run, the same internal loading control (one of the samples) was added to each gel and bands were normalised against this value.

Statistical analysis was performed using MiniTab on a PC using analysis of variance (Kruskal Wallis for non-parametric data and ANOVA for normally distributed data). Comparison of groups was performed by the Mann Whitney test. The strength of relationship between two variables was tested using Spearman rank correlation. *p*<0.05 was considered to be statistically significant.

### Patients recruited to determine whether APJ mRNA expression excised from cyanotic patients differs from control (acyanotic) patients after exposure to 15–30 min ischemia

Due to the small amount of tissue obtained from each patient a new group of patients were recruited for this experiment. Myocardial tissue samples were collected from cyanotic and control patients during corrective heart surgery and processed as outlined above. Collection continued until a minimum of 5 patients were in each group (according to original power calculations). In the end twelve patients were recruited (Table 2). Seven patients were cyanotic and were comprised of TOF patients (RV muscle resection). Five patients were used as controls (acyanotic) patients, comprising of sub-aortic stenosis (left V muscle resected) and truncus arteriosus (TA) patients (RV muscle resection). Myocardial tissue was collected in theatre, transferred immediately to RNA*later* and stored overnight at 4°C to stabilize the RNA. Samples from both groups were collected between 15–30 min after initiation of the cross-clamp. This removed any variability in mRNA due to variations in timing of sample collection.

**Table 2:** Patients recruited for experiment to determine whether APJ mRNA expression in myocardium excised from cyanotic patients differs from control (acyanotic) patients.

Patient Group	O_2_ Saturation	Gender	Age (months)
TOF	Cyanotic	Female	1 3
TOF	Cyanotic	Male	1 4
TOF	Cyanotic	Male	1 4
TOF	Cyanotic	Male	11
TOF	Cyanotic	Female	12
TOF	Cyanotic	Male	11
Fallot variant	Cyanotic	Female	3
Sub-aortic stenosis	Acyanotic	Male	7
Sub-aortic stenosis	Acyanotic	Female	148
Sub-aortic stenosis	Acyanotic	Male	32
Truncus arteriosus	Acyanotic	Male	1
Sub-aortic stenosis	Acyanotic	Female	11

### RNA extraction

The next day RNA was extracted from the tissue stored in RNA*later* using the RNeasy Fibrous Tissue Midi Kit (Qiagen, cat. no. 75742). Once RNA was successfully eluted in RNase free water, the RNA concentration (ng/µl) and purity was then determined using a NanoDrop (Thermo Scientific). The RNA was then stored in aliquots at −80°C.

### Reverse transcription (RT) of mRNA

For the RT reaction mRNA was removed from −80°C storage and kept at 4°C. Using the QuantiTect Reverse transcription Kit (Qiagen, 205310) and GoScript reverse transcriptase (Promega, A5003) the RNA was reverse transcribed into cDNA. The products of the PCR reaction were separated on a 2% agarose gel alongside a 100 bp ladder (Sigma-Aldrich, P1473). The quality of the cDNA was checked with the Human cDNAOK kit (Microzone, 2HCDOK-150).

### Primers

The APJ receptor primer sequences (custom made, Sigma U.K.) produced a 89 base pair amplicon [17]. The primers (forward CTATCCTGTTTTCTGAGTGTGAGG; reverse-CTAAGGGCTGGAGCACTAATTATC were checked to ensure they met the criteria for RT-PCR (http://www.bioinformatics.nl/cgibin/primer3plus/primer3plus.cgi);(https://ngrl.manchester.ac.uk/SNPCheckV2/snpcheck.htm); (http://www.ncbi.nlm.nih.gov/projects/epcr/reverse.cgi);http://www.sigma-genosys.com/calc/DNACalc.asp). A 100 µM primer stock solution was made. From this, a 5 µM working solution of each primer was made. This concentration of working primer stock was based on optimisation experiments for the endpoint and qPCR machine used. Both the stock and primer stock solution were stored at −20°C. Quantitative RT-PCR was performed using the GoTaq qPCR Master Mix (Promega, A6001) and the StepOnePlus qPCR machine (Applied Biosystems). The endogenous control used was β-Actin (primers designed in-house): Forward primer – GCGGGAAATCGTGCGTGACATT and reverse primer – GATGGAGTTGAAGGTAGTTTCGTG, amplicon size −232 base pairs. The experiments were performed using Microamp fast optical 96 well plates (Applied Biosystems, 4346906) using the following program: Holding stage − 95°C for 20 sec, Cycling stage −95°C for 3 sec, 60°C for 30 seconds ×50 cycles, Melt curve 95°C for 15 sec, 60°C for 1 min, 95°C for 15 sec.

Differences in gene expression were calculated using the Comparative Ct method [18] to give RQ of gene expression using the Stepone Software v2.1 (Applied Biosystems). Statistical analysis was performed using GraphPad Prism 6 Software©. The data did not follow a normal distribution therefore non-parametric (Mann-Whitney U test) statistical analysis was undertaken. A p-value of <0.05 (two-tailed) was considered statistically significant.

### Does reperfusion of myocardium with different oxygen concentration affect APJ receptor expression?

During open-heart surgery with CPD, the myocardium is rendered ischemic. Reperfusion, performed at super-physiological oxygen levels, may result in an ischemic-reperfusion insult to the myocardium. This in turn may activate protective mechanisms. Thus the aim of this experiment was to expose ischemic myocardium, taken from patients undergoing corrective cardiac surgery, to 2% O_2_ (hypoxia), 20% O_2_ (normoxia) and 60% O_2_ (hyperoxia) *in vitro* (to mimic reperfusion that occurs during paediatric open-heart surgery) and then determine the effects on APJ receptor mRNA expression. Again due to limited tissue new patients were recruited (Table 3). Samples power required fewer patients since the patient's own sample was split for *in vitro* analysis. Myocardium was collected in theatre, placed into culture media which had been pre-gassed to 2% O_2_ (ischemia), and immediately transported to the adjacent laboratory. The sampling time, between 15–30 min following initiation of the cross-clamp, ensured all samples were collected within a similar time range. Two NuAire incubators were set at 2%O_2_/5%CO_2_/93%N_2_ (hypoxia) and 20%O_2_/5% CO_2_/75%N_2_ (normoxia). A third incubator (New Brunswick 48R carbon dioxide (CO_2_) incubator) was used to achieve the maximum possible level of hyperoxia (60%O_2_/5%CO_2_/35%N_2_). To mimic reperfusion, the samples were quickly cut into equal size pieces and followed one of three treatments: they were placed into culture flasks containing media that had been pre-equilibrated to 2%, 20% or 60% oxygen. The flasks were then placed into the appropriate incubator and maintained for a further 4 h. The 4 h time point was chosen following a review of the literature [19] for optimal times for mRNA induction. At the end of the incubation, tissue was removed and immediately processed for RNA extraction and APJ receptor expression as described above. Statistical analysis was performed for paired analysis using GraphPad Prism 6 Software©. The data did not follow a normal distribution therefore non-parametric statistical analysis was undertaken using the Mann-Whitney U test. A p-value of <0.05 (two-tailed) was considered as statistically significant. All graphs are shown as box and whiskers plots. The bottom and top box are the first and third quartiles. The centre line is the median. The whiskers represent the lowest and highest values.

**Table 3:** Patients recruited for experiment to determine the effect of re-perfusing myocardium at different O_2_ concentrations *in vitro* on APJ mRNA expression.

Patient Group	Cyanotic state	Gender	Age (months)
TOF	Cyanotic	Male	72
TOF	Cyanotic	Male	10
TOF	Cyanotic	Female	16
TOF	Cyanotic	Female	6
TOF	Cyanotic	Male	11
Complex TOF	Cyanotic	Male	60
Redo TOF	Acyanotic	Female	77
Ventricular septal defect	Acyanotic	Female	14
Sub-Aortic obstruction	Aycanotic	Male	15
Truncus Arteriosus	Acyanotic	Male	1

## Results

### Western Blot Analysis

To date the APJ receptor has not been identified in the infant myocardium. Figure 1a shows one representative Western blot of some of the patient samples. A 60 kDa band, known to be the size of the N-glycosylated APJ receptor [20] was identified in all of the patient samples. Not surprisingly, as is often the case when sampling patient groups such as the one in this study, the amount of receptor differed between individuals. Analysis of the same samples for constitutively expressed HSP 70 showed expression was similar in all samples supporting our previous observation that HSP 70 does not vary significantly between patients. Thus the differences in AJP between patients was not due to differences in the amount of total protein in each aliquot but reflects the fact that AJP receptor varies between individuals.

**Figure 1:** **1a**: Western blot analysis of APJ receptor expression. Upper blot shows APJ receptor expression in myocardium obtained from patients used in the study. The lower blot shows HSP 70 levels in the same patient samples Numbers identify individual patients. C is internal placental loading control added to all gels. 50 µg protein was loaded in all wells. **Figure 1b**: APP receptor analysis in relation to length of the surgical time. Box and whiskers plot shows APJ receptor in the myocardial samples collected at the start of surgery (<10 min) and samples collected after 10 min until the end of surgery.

Figure 1b shows that expression of the APJ receptor in the samples collected after 10 min until the end of surgery was increased compared to the samples at the start of surgery (<10 min) (p<0.05). This division allowed equal numbers of samples to be studied and to allow a time that was very close to the start of surgery versus samples taken later. Therefore as time of cardioplegia and ischemia increased so, overall, did expression of the APJ receptor. Clearly there is overlap between the two times intervals studied and there is some variability as expected from human studies; nonetheless the fact that protein levels alter relatively quickly after the 10 min time point suggest this may be more likely due to stabilisation of APJ rather than new protein synthesis however this question cannot be answered in the current study.

Oxygen extraction ratio is an indicator of the adequacy of cardiac output in the early post-operative phase calculated from the oxygen content of systemic arterial and mixed venous blood samples. There was no significant association between O_2_ extraction ratio and APJ receptor expression in myocardial samples collected <10 min. There was however a significant association between O_2_ extraction ratio and APJ receptor expression in samples collected >10 minute with higher APJ receptor expression associated with lower oxygen extraction ratio (p = 0.021, rho = −0.523).

Mixed venous oxygen saturation (SvO_2_) is a measure of the O_2_ saturation of the venous blood taken from the right atrium or pulmonary artery, representative of O_2_ saturation for the entire venous circulation. It reflects the balance between oxygen delivery and tissue consumption and acts an indicator of cardiac output. When the APJ receptor expression in samples taken >10 minutes was correlated to SvO_2_ there was a significant positive correlation with higher APJ levels associated with a higher SvO_2_ (p = 0.028, rho 0.52). Again this association was not present for samples collected <10 minutes.

There were no other correlations between APJ receptor expression and any of the other clinical parameters listed in Table 1.

### RNA results

The next set of experiments was to determine if APJ expression in myocardium excised from cyanotic patients differ from control (acyanotic) patients. The results are shown in Figure 2. There was no difference in APJ receptor expression between both groups.

**Figure 2:** APJ receptor analysis for cyanotic and acyanotic groups. Comparison of myocardial APJ receptor mRNA for the cyanotic (n = 7) and acyanotic (n = 5) patient groups shown in Table 2. Expression was calculated using the Comparative Ct method to give RQ of gene expression using the StepOne Software v2.1). Statistical analysis was performed using the Mann-Whitney U test. Data shown as box and whiskers plot.

The third and final set of experiments was to determine if reperfusion of myocardium with different oxygen concentration affected APJ receptor mRNA expression. The results are show in Figure 3. No significant differences were found between groups. A further paired analysis was performed to compare the results from samples obtained from cyanotic patients compared to acyanotic patients. There was no difference between cyanotic and acyanotic patient samples in their response to re-oxygenation (Figure 4).

**Figure 3:** Comparison of myocardial APJ receptor mRNA for samples collected from patients shown in Table 3 then re-perfused at 2, 20 or 60% O_2_ for 4 h. Baseline are samples analysed before the re-perfusion experiments started. Expression was calculated using the Comparative Ct method to give RQ of gene expression using the StepOne Software v2.1). Statistical analysis was performed using the Mann-Whitney U test. Data shown as box and whiskers plot.

**Figure 4:** Comparison of myocardial APJ receptor mRNA for samples collected from patients shown in Table 3 then re-perfused at 2, 20 or 60% O_2_ for 4 h. The same patients as for Table 3 were use but split into 2 groups (cyanotic and acyanotic). Expression was calculated using the Comparative Ct method to give RQ of gene expression using the StepOne Software v2.1). Statistical analysis was performed using the Mann-Whitney U test. Data shown as box and whiskers plot.

## Discussion

This is the first study to have shown evidence of APJ receptor expression in the early, immature myocardium. The expression and function of Apelin-APJ in the adult heart and its role in heart failure has been investigated [8], [9], [21]–[23] but expression and function has not been investigated in the context of paediatric cardiac surgery for congenital heart defect repair. Western blot analysis of the APJ receptor produced evidence that the APJ receptor is expressed in the RV of the immature myocardium.

As a result of the theoretical advantageous effects of Apelin-APJ function, much of the research into Apelin and receptor-mediated effects have been focused on heart failure. Expression of Apelin and APJ in the myocardium is increased in response to heart failure in rats [20] and this may be part of a compensatory mechanism in an attempt to restore normal cardiac output. Apelin may protect the heart against fibrotic remodelling [24], which contributes to the pathogenesis of heart failure. There have been positive results from one of the few human studies in which heart failure patients were infused with Apelin and demonstrated improved cardiac output and concomitant peripheral and coronary vasodilation [12]. As heart failure progresses and ventricular dysfunction worsens, myocardial Apelin production is reduced [8] and Apelin infusion reduced infarct size after coronary artery occlusion in rodents [25]. The APJ receptor is also expressed in higher levels in mature coronary vessels after prolonged periods of ischemia [23]. Apelin production is also mediated through hypoxia [26]. Rodent models have shown direction protection against IR injury by Apelin administration and it has been proven that Apelin reduces this damage by reducing endoplasmic reticulum stress and therefore attenuating ER-dependent apoptosis via the APJ receptor [27].

Previous studies on liver cells have shown that the APJ receptor is up-regulated in response to hypoxia [17]. For the first time we have shown that for myocardium resected during ischemic period of surgery, those samples that are exposed too longer duration of ischemia express higher levels of APJ receptor. These findings support but do not prove the hypothesis that ischemic conditions upregulate expression of APJ in the myocardium as part of a cardioprotective mechanism or alternatively prevent breakdown/turnover of existing receptors. Depending on the apelin fragments produced *in vivo*, the apelin receptor may be stabilized in different conformational states. This was demonstrated by functional dissociation of apelin receptor signaling and endocytosis resulting in different depressor responses [28]. Further experiments in this area are however warranted.

Oxygen extraction ratio is the difference between arterial and venous O_2_. A low oxygen extraction ratio reflects better cardiac output. In this study a low oxygen extraction ratio correlated with higher amounts of APJ receptor in the samples collected after 10 min only. Again these findings also support a protective effect of the APJ receptor as the surgical time progresses perhaps due to the known effects of receptor activation (inotropy, peripheral vasodilation and diuresis).

APJ expression in the period of surgery after 10 min correlated with increased mixed venous oxygen saturations [SvO_2_]. SvO_2_ is another surrogate maker of cardiac output in the post-operative phase, with low venous saturations indicating reduced oxygen delivery to the peripheral tissues. Taken together, the relationship between both oxygen extraction ratio and mixed venous oxygen saturations and APJ expression (>10 min) would suggest increased APJ expression reduces the decrease in cardiac output observed early after surgery. Therefore one explanation is that myocardium, with the ability to increase APJ expression during the ischemic period, may be better protected against ischemic-reperfusion injury with subsequent improved post-operative contractility. However we did not observe any relationship between APJ and echocardiographic parameters of contractility. Whether any relationship might exist in subsequent weeks or months or whether more subtle measurements of contractility may detect a relationship would require further investigation.

Troponin is a standard biomarker of cardiac stress and damage and it has been postulated that Apelin can be used as a marker for myocardial damage in a similar way to Troponin, such as in myocardial infarction [29]. Serum Apelin has been correlated with Troponin levels in patients with acute coronary syndrome [29]. In the present study there was no correlation between APJ expression and post-operative day one serum Troponin levels. A future study measuring serum Apelin in these patients would be of interest.

Conclusions and limitations: Cyanotic versus acyanotic patients: Although the age range of patients used appeared wide this can be explained by one outlier, one patient at 148 months. When this patients was removed from the analysis the results for APJ did not change nor was there any correlation with age. As far as LV/RV sampling, only one patient had LV muscle resected. Removing this patient from the analysis did not alter the findings. Similarly for the re-perfusion experiments at different oxygen concentrations one case was LV. Removing this patient did not alter the findings. In the comparison between cyanotic and acyanotic patients the patient cohort differ. Clearly there are many patient groups that could be compared however this study provides the first investigation into the comparison of the Apelin receptor in the setting of paediatric heart surgery and future studies are warranted”

It would also be interesting in future studies to differentiate between BT shunt and non-BT shunt patients and then differentiating on the degree of right ventricular outflow tract obstruction as well as right atrial as Apelin may be expressed more from atrium than from ventricle.”

Studies using human/infant myocardium are limited by the tiny amount of tissue that is available. RT-PCR allows analysis of the APJ receptor on very small pieces of tissue. Had changes been observed then a follow up study on protein analysis may have been justified. Samples of myocardium resected for this project were primarily from the RV or right ventricular outflow tract. It is not known whether expression of APJ receptor in these areas are representative of the rest of the immature heart and specifically the left ventricle. It is however the RV which is most at risk of post-operative dysfunction in TOF and therefore the most appropriate area of the myocardium to measure APJ expression as affected by the surgery. The number of patients available also make studies such as this very difficult to do yet it is important that they are done to understand the human situation. There are no previous studies similar to this however we were able to power the experiments based on our previous studies on myocardium and *in vitro* re-oxygenation experiments on placental explants [30]–[31].

The known physiological functions of Apelin-APJ have made it a focus for treatment in the context of heart failure [8], [9], [12], [21], [22]. Successful clinical trials [12] and development of a non-peptide APJ receptor agonist [32] suggest that modulation of the APJ receptor system is a possibility in heart failure therapy. The possibility that Apelin administration or methods to modulate the APJ receptor could be considered in the context of congenital heart defects and prophylactic cardioprotection for surgical repair involving cardiopulmonary bypass may one day prove to be beneficial although much research is still required.
